# RANKL/RANK/OPG system beyond bone remodeling: involvement in breast cancer and clinical perspectives

**DOI:** 10.1186/s13046-018-1001-2

**Published:** 2019-01-08

**Authors:** Marco Infante, Alessandra Fabi, Francesco Cognetti, Stefania Gorini, Massimiliano Caprio, Andrea Fabbri

**Affiliations:** 1 Unit of Endocrinology and Metabolic Diseases, Department of Systems Medicine, CTO A. Alesini Hospital, ASL Roma 2, University Tor Vergata, Via San Nemesio, 21, 00145 Rome, Italy; 2 Division of Medical Oncology 1, Regina Elena National Cancer Institute, Via Elio Chianesi, 53, 00144 Rome, Italy; 3 Laboratory of Cardiovascular Endocrinology, IRCCS San Raffaele Pisana, Via di Val Cannuta, 247, 00166 Rome, Italy; 4 Department of Human Sciences and Promotion of the Quality of Life, San Raffaele Roma Open University, Via di Val Cannuta, 247, 00166 Rome, Italy

**Keywords:** RANKL, RANK, OPG, Mammary gland, Breast tumorigenesis, Breast cancer, Metastatic bone disease, RANKL inhibition, Adjuvant Denosumab

## Abstract

RANKL/RANK/OPG system consists of three essential signaling molecules: i) the receptor activator of nuclear factor (NF)-kB-ligand (RANKL), ii) the receptor activator of NF-kB (RANK), and iii) the soluble decoy receptor osteoprotegerin (OPG). Although this system is critical for the regulation of osteoclast differentiation/activation and calcium release from the skeleton, different studies have elucidated its specific role in mammary gland physiology and hormone-driven epithelial proliferation during pregnancy. Of note, several data suggest that progesterone induces mammary RANKL expression in mice and humans. In turn, RANKL controls cell proliferation in breast epithelium under physiological conditions typically associated with higher serum progesterone levels, such as luteal phase of the menstrual cycle and pregnancy. Hence, RANKL/RANK system can be regarded as a major downstream mediator of progesterone-driven mammary epithelial cells proliferation, potentially contributing to breast cancer initiation and progression. Expression of RANKL, RANK, and OPG has been detected in breast cancer cell lines and in human primary breast cancers. To date, dysregulation of RANKL/RANK/OPG system at the skeletal level has been widely documented in the context of metastatic bone disease. In fact, RANKL inhibition through the RANKL-blocking human monoclonal antibody denosumab represents a well-established therapeutic option to prevent skeletal-related events in metastatic bone disease and adjuvant therapy-induced bone loss in breast cancer. On the other hand, the exact role of OPG in breast tumorigenesis is still unclear. This review focuses on molecular mechanisms linking RANKL/RANK/OPG system to mammary tumorigenesis, highlighting pre-clinical and clinical evidence for the potential efficacy of RANKL inhibition as a prevention strategy and adjuvant therapy in breast cancer settings.

## Background

The RANKL/RANK/OPG system was first identified in the late-1990s as a pivotal regulator of bone remodeling [1–3]. It consists of three main signaling molecules: the cytokine receptor activator of nuclear factor (NF)-kB-ligand (RANKL; see Table 1 for the list of abbreviations), the receptor activator of NF-kB (RANK), and the soluble decoy receptor osteoprotegerin (OPG). RANKL, formerly identified as TRANCE (TNF-related activation-induced cytokine) [4], is a tumor necrosis factor (TNF) family member expressed by bone marrow stromal cells, osteocytes and osteoblasts [3]. RANKL is a homotrimeric transmembrane protein typically expressed on osteoblasts and activated T cells, although it can be also produced as a secretory protein [5]. RANKL binds to its signaling receptor RANK - a tumor necrosis factor receptor (TNFR) family member - on the surface of osteoclast precursor cells, leading to the fusion of these cells into multinucleated cells which then differentiate into mature osteoclasts [2, 6, 7]. Mature osteoclasts adhere to bone surface and promote bone resorption by secreting acid and lytic enzymes (e.g. cathepsin K, tartrate-resistant acid phosphatase) [2, 8]. OPG is primarily expressed by bone marrow stromal cells and osteoblasts, and represents an atypical member of the TNFR family, since it functions as a soluble decoy receptor lacking a transmembrane domain [3, 9]. OPG has been found to bind RANKL with approximately 500-fold higher affinity than RANK [10]. Hence, OPG prevents RANKL from binding to its receptor RANK, inhibiting osteoclastogenesis and protecting the bone from excessive osteoclast-mediated resorption [11, 12].

**Table 1:** List of abbreviations

*BRCA1*	Breast cancer susceptibility gene 1
*BRCA2*	Breast cancer susceptibility gene 2
CRAd	Conditionally replicating adenovirus
DMBA	7,14-dimethylbenz[a]anthracene
EGF	Epidermal growth factor
EGFR	Epidermal growth factor receptor
ELISA	Enzyme-linked immunosorbent assay
EMT	Epithelial-mesenchymal transition
ER	Estrogen receptor
ErbB	Epidermal growth factor receptor
ErbB2	Epidermal growth factor receptor 2
HRT	Hormone replacement therapy
Id2	Inhibitor of DNA binding protein 2
IkB	Inhibitor of kappa B
IkBα	Inhibitor of kappa Bα
IKK-α	Inhibitor-kB kinase-α
IgG	Immunoglobulin G
IHC methods	Immunohistochemical methods
IL-1	Interleukin-1
IL-6	Interleukin-6
IL-8	Interleukin-8
Jak2	Janus kinase 2
LECs	Luminal epithelial cells
MaSCs	Mammary stem cells
M-CSF	Macrophage colony-stimulating factor
MECs	Myoepithelial cells
MMTV	Mouse mammary tumor virus
MPA	Medroxyprogesterone acetate
NF-kB	Nuclear factor-kB
OPG	Osteoprotegerin
PCR	Polymerase chain reaction
PR	Progesterone receptor
PRLR	Prolactin receptor
PTHrP	Parathyroid hormone-related protein
RANK	Receptor activator of NF-kB
RANKL	Receptor activator of NF-kB-ligand
SREs	Skeletal-related events
STAT5a	Signal transducer and activator of transcription 5a
TGF-β	Transforming growth factor-β
TNBC	Triple-negative breast cancer
TNF	Tumor necrosis factor
TNFR	Tumor necrosis factor receptor
*TNFRSF11A*	TNF Receptor Superfamily Member 11a
TNF-α	Tumor necrosis factor-α
TRAF	TNF receptor-associated factor
TRAF2	TNF receptor-associated factor-2
TRAIL	TNF related apoptosis-inducing ligand
TRANCE	TNF-related activation-induced cytokine

However, over the last two decades RANKL/RANK axis has been identified as a critical signaling pathway involved in several mechanisms beyond bone homeostasis [13]. Specifically, it is essential for different processes affecting immune regulation, such as interaction between T cells and dendritic cells [14], lymphocyte development, lymph node organogenesis [15], and thymic development [16]. Furthermore, various alternative splicing-derived isoforms of RANKL and RANK have been detected [17–20], suggesting a more complex role of RANKL/RANK system than previously thought. Ikeda et al. identified two additional isoforms of RANKL, namely: i) RANKL 2, with a shorter intracellular domain than the original form (RANK 1), and ii) RANKL 3, which lacks a transmembrane domain and represents a putative soluble form. The three isoforms are differentially expressed and finely regulated in several cell lines (bone marrow stromal cells, preosteoblastic cells, and various T cells subsets), suggesting the existence of multiple tissue-specific pathways with specific roles in osteoclastogenesis and T cell differentiation [17].

Intriguingly, RANKL/RANK axis is also required for hormone-driven mammary gland development during pregnancy [21]. Given the proliferative effect of RANKL/RANK signaling on mammary epithelial cells, several studies suggested a potential involvement of RANKL/RANK system in breast cancer initiation and metastatic progression [22–29]. Conversely, data on the role of OPG in breast physiology and tumorigenesis are less univocal and require more investigations [30–36]. This narrative review is focused on the emerging roles of RANKL/RANK/OPG system in mammary gland pathophysiology, highlighting therapeutic potential of this pathway in human breast cancer.

## RANKL/RANK/OPG system and mammary gland development

Different studies elucidated the central role of RANKL/RANK system in mammary gland physiology and hormone-driven epithelial proliferation during pregnancy [3, 21, 22, 37–41]. In mammals, mammary gland represents a vital organ required to provide maternal nourishment to newborns in form of calcium-enriched milk. Therefore, it is likely that during evolution RANKL/RANK/OPG system - originally required only for bone remodeling - shifted to calcium-related functions even in mammary gland [21]. The mammary epithelium is made of an inner layer of luminal epithelial cells (LECs) and an outer layer consisting of myoepithelial cells (MECs) adjacent to a basement membrane that separates it from the underlying mammary stroma [42]. LECs form the lining of ducts/alveoli and are involved in milk synthesis and secretion during lactation, whereas MECs are smooth muscle-like contractile cells facilitating excretion of milk from the mammary gland [43]. Ductal tree development during sexual maturation and alveologenesis throughout pregnancy/lactation both require coordinated morphogenesis and proliferation of LECs and MECs [39]. In this context, evidence from murine models supports that RANKL is a key regulator of mammary epithelial cells proliferation and differentiation, driving the morphogenesis of a lactating mammary gland during pregnancy [21]. Accordingly, RANKL expression can be induced in murine mammary epithelial cells after exposure to pregnancy hormones, such as progesterone, prolactin and parathyroid hormone-related protein (PTHrP) [21, 44]. This suggests that RANKL is a major effector of hormone-driven mammary epithelium response during early pregnancy [21]. In fact, RANKL is absent in virgin mammary glands, but its expression progressively increases in LECs between the 17th and 26th day of the menstrual cycle [21], and throughout pregnancy [38]. On the other hand, RANK is present at low levels in both luminal and basal mammary epithelial cells, but its expression is higher at mid-gestation (especially at the level of ductal branch points) [45]. Genetic studies documented that both RANKL and progesterone receptor (PR) are localized in LECs, acting on similar stages of the mammary gland morphogenesis [44]. Notably, progesterone has mitogenic effects on mammary epithelial cells through two distinct waves of proliferation. The first wave affects PR-positive cells and requires cyclin D1, while a second larger wave encompasses PR-negative cells and relies on RANKL. In particular, progesterone upregulates RANKL expression on PR-positive LECs. In turn, RANKL drives proliferation of neighboring estrogen receptor (ER)/PR-negative LECs, acting in a paracrine fashion via its receptor RANK [23, 40, 46] (see Fig. 1a). Indeed, mice lacking PR-B isoform show defects of ductal side-branching and lobulo-alveologenesis during pregnancy, along with impaired RANKL expression [47]. Conversely, ectopic expression of RANKL completely blunts defects of PR-deficient cells in the morphogenesis of lactating mammary gland, supporting a crucial role of RANKL in mediating progesterone-driven mitogenic effects on mammary epithelial cells [40, 41]. Moreover, it has been found that RANKL is able to increase proliferation of MECs in cultured mammary organoids obtained from adult mice [39] (Fig. 1a). Similar to progesterone, prolactin is also necessary for a proper development of mammary gland during pregnancy. Specifically, prolactin acts through Jak2/STAT5a signaling in order to induce RANKL expression by mammary epithelial cells [38]. Altogether, these findings highlight the existence of a strict relationship between progesterone, prolactin and RANKL/RANK system in driving the morphological changes of mammary gland during pregnancy.

**Fig. 1:** Schematic diagram showing PR/RANKL pathway and downstream RANK-mediated signaling in mammary epithelial cells. **a** Natural or synthetic progesterone binds to its receptor in PR-positive breast luminal cell, leading to an increase in RANKL protein levels mainly through stabilization of its mRNA. Then, RANKL binds to its cognate receptor RANK expressed on the surface of the neighboring PR-negative breast luminal cell, activating downstream signaling pathways that promote cell proliferation. Basal cells (MECs and MaSCs, drawn in green at the bottom of the figure) constitutively express RANK on their surface, but they lack PR. RANKL produced by PR-positive breast luminal cells further up-regulates RANK expression on MECs and MaSCs surface, and activates RANK-downstream signaling pathways promoting cell proliferation, expansion and survival. **b** RANK-IKK-α-NF-kB-cyclin D1 pathway (1), and RANK-Id2-p21 pathway (2) represent the two main signaling pathways activated by RANK in mammary epithelial cells. IKK-α catalyzes phosphorylation, ubiquitination and proteasome degradation of IkBα, leading to its dissociation from NF-kB, which then migrates to the nucleus and induces *cyclin D1* transcription. On the other hand, Id2 translocates into the nucleus and reduces expression of the cell cycle inhibitor p21. Altogether, these molecular events result in increased proliferation and survival of mammary epithelial cells. RANK-c is a RANK isoform derived from alternative splicing of *RANK* gene, which has been identified in breast cancer cell lines and breast tumors. It acts as a dominant negative regulator of RANK-dependent NF-kB activation, inhibiting the NF-kB-mediated cell survival effect and correlating with lower cell motility and proliferative index. RANK-c may exert its function through the intracellular interaction with other key molecules, such as TRAF2 and EGFR. Notably, RANK-c has also been shown to act as a negative regulator of EGFR signaling, inhibiting EGFR phosphorylation after EGF ligand stimulation. Abbreviations: EGF, Epidermal growth factor; EGFR, Epidermal growth factor receptor; Id2, inhibitor of DNA binding protein 2; IkBα, inhibitor of kappa Bα; IKK-α, inhibitor-kB kinase-α; LECs, luminal epithelial cells; MaSCs, mammary stem cells; MECs, myoepithelial cells; NF-kB, nuclear factor-kB; Pg, natural or synthetic progesterone; PR, progesterone receptor; RANK, receptor activator of NF-kB; RANKL, receptor activator of NF-kB-ligand; TRAF2, TNF receptor-associated factor-2

At a molecular level, RANKL binds RANK - constitutively expressed on the surface of basal and luminal mammary epithelial cells - and regulates proliferation of mammary epithelial cells. RANKL/RANK axis functions through two different downstream signaling pathways: 1) the first pathway triggers activation of inhibitor-kB kinase(IKK)-α, resulting in proteasome degradation of IkBα (inhibitor of kappa Bα) and its dissociation from NF-kB, which migrates to the nucleus and induces *cyclin D1* transcription [48–50]; 2) the second pathway promotes nuclear translocation of the transcriptional regulator inhibitor of DNA binding protein 2 (Id2), which subsequently downregulates cell cycle inhibitor p21 [51] (see Fig. 1b). These molecular pathways provide survival and proliferative signals required for development of lobulo-alveolar structures during the course of pregnancy [48, 52]. Accordingly, RANKL and RANK null mice exhibit normal mammary fat pad development during puberty, but they show impaired lobulo-alveolar morphogenesis during pregnancy and lactational defect at parturition due to increased apoptosis and defective proliferation of mammary epithelium [21]. In agreement with these findings, female mutant mice lacking PR, prolactin receptor (PRLR), IKK-α, Id2, or STAT5a display similar phenotypes to those observed in RANKL or RANK-deficient mice [47, 48, 53–55]. Conversely, transgenic mice overexpressing RANKL or RANK show increased proliferation of mammary epithelium, with precocious ductal-side branching and alveolar budding [45, 54]. Importantly, RANKL/RANK axis is also involved in mammary stem cell biology [56, 57]. RANKL has been identified as a paracrine effector of progesterone-driven expansion of adult mammary stem cells (MaSCs) observed during pregnancy and luteal phase of the menstrual cycle. MaSCs reside in the basal compartment of mammary epithelium and have the ability of self-renewal and multipotency. In fact, MaSCs can differentiate into all mammary cell lineages (ductal and alveolar LECs, as well as ductal and alveolar MECs), being able to regenerate the entire mammary epithelial tree [58, 59]. Although MaSCs lack both ER and PR, they are highly responsive to steroid hormone signaling, as supported by the fact that MaSCs pool increases during the luteal diestrus phase and throughout pregnancy [56, 57]. Progesterone promotes selective upregulation of RANKL and RANK on breast luminal and MaSC-enriched basal cells, respectively. RANKL from LECs binds to its cognate receptor RANK on basal cells, further upregulating RANK expression and activating RANK downstream signaling pathways that promote MaSCs proliferation and expansion [56, 57, 60] (Fig. 1a). Accordingly, Joshi et al. examined murine models treated with a RANKL inhibitor, documenting that loss of RANK signaling blunts the progesterone-induced proliferation of hormone receptor-negative murine mammary progenitors [61]. Moreover, whole-body anti-RANKL treatment of virgin and pregnant mice significantly impairs the clonogenicity of MaSC-enriched basal cell population in vitro [56]. In addition, selective genetic ablation of RANK in the basal compartment of mammary epithelium leads to defective lobulo-alveolar development and lactation [25], while no defect is observed when RANK deletion occurs in luminal cells [62]. These findings highly suggest that RANK signaling is crucial in basal cells - but not in luminal cells - for the development of lactating mammary tissue, and RANKL/RANK axis promotes progesterone-induced MaSCs expansion in a paracrine fashion during the luteal phase of the menstrual cycle and throughout pregnancy.

In order to assess whether RANKL plays all the aforementioned physiological roles also in humans, Tanos et al. developed an ex vivo model consisting of tissue microstructures isolated from fresh human breast tissue specimens of healthy donors [63]. Of note, PR signaling has been shown to promote LECs proliferation by induction of the same mediators of progesterone action identified in murine models, namely Wnt-4 and RANKL [40, 63, 64]. Specifically, progesterone controls RANKL mRNA levels predominantly by post-transcriptional mechanisms (increased mRNA maturation/stability) [63]. RANKL protein expression is also positively associated with serum progesterone concentrations in the human breast in vivo [63]. Accordingly, Azim et al. found that pregnancy increases RANKL expression both in normal human breast and primary breast tumors [65]. These data suggest that progesterone-induced RANKL expression may represent a conserved hormonal pathway in mice and humans, able to control cell proliferation in breast epithelium under physiological conditions commonly associated with higher serum progesterone levels (e.g. luteal phase of the menstrual cycle, pregnancy).

On the other hand, data on the exact role of OPG in mammary gland physiology are not univocal. Even though OPG mRNA is expressed in normal breast tissue and its transcription is regulated by pregnancy hormones (especially estrogen) [66], there is scarce evidence for a direct role of OPG in breast development and function [30]. In fact, neither female OPG-overexpressing transgenic mice nor OPG-deficient mice show any impairment in mammary gland formation [32, 33]. On the other hand, Vidal et al. detected 1000-fold higher concentrations of OPG in human milk than in serum, suggesting a possible role of OPG in mammary gland development during lactation. The same study showed that both human breast milk cells and human mammary epithelial cell line MCF-7 express OPG [34]. However, these findings still do not demonstrate an essential role of OPG in breast development and pregnancy-related mammary gland morphogenesis, and studies elucidating the role of OPG in breast physiology are awaited.

## Role of RANKL/RANK system in breast tumorigenesis

Breast cancer represents the most common female cancer, accounting for around 25% of all cancers [67]. Risk factors for breast cancer include age over 40, genetic predisposition, Caucasian race, early menarche, late menopause, late childbearing, hormonal contraception, and hormone replacement therapy (HRT) [68]. Progesterone and its synthetic derivatives (progestins) are commonly used in combined HRT (estrogen plus progesterone) and hormonal contraception [69, 70]. The Women’s Health Initiative and the Million Women Study provided evidence that women using combined HRT show a significant increase in risk of incident and fatal breast cancer, compared with women using estrogen alone [71–73]. Other studies documented that risk for breast cancer development is associated with menstrual cycles and related peaks in serum progesterone levels [74]. Overall, progesterone and progestins are considered key factors for increased breast cancer risk in women. Several pre-clinical studies demonstrated that RANKL/RANK system promotes breast tumorigenesis [23, 24, 26, 27, 46], suggesting that such system may account, at least in part, for the increased incidence of breast cancer associated with use of progesterone and progestins. As previously mentioned, progesterone is a powerful driver of RANKL expression, which in turn induces proliferation of mammary epithelial and stem cells both in mice and humans [40, 46, 63, 75]. Intriguingly, breast tumorigenesis is sustained through the same pathway. First, the expression of RANKL and RANK has been documented in breast cancer cell lines and in human breast cancers [23, 24, 76–78]. Moreover, RANK expression in tumor tissue has been significantly associated with poor disease-free survival in primary human breast cancer [78]. A growing body of evidence indicates that RANKL/RANK axis is a crucial mediator of the proliferative changes observed in mammary epithelium during the onset of primary progesterone-driven breast cancer [23, 25, 79]. Schramek et al. showed that female mice treated with the progestin medroxyprogesterone acetate (MPA) exhibit a massive upregulation of RANKL expression in mammary epithelial cells, resulting in a rapid and marked cell proliferation that is instead significantly decreased in RANK deficient mice [25]. Given that MPA-induced tumorigenesis requires a carcinogen [80], the authors used the DNA-damaging agent 7,14-dimethylbenz[a]anthracene (DMBA) in combination with MPA to promote DNA mutations and mammary cancer development [25]. Surprisingly, RANK-deficient mice showed a remarkable delay in the onset of MPA/DMBA-induced mammary cancer, as well as an enhanced survival when compared with the wild-type controls. Similarly, IKK-α knockout mice exhibited a delayed onset of mammary tumors after MPA/DMBA treatment, indicating that RANKL/RANK system acts through IKK-α pathway even in hormone-driven mammary tumorigenesis [25]. Another study reported that transgenic mice with a gain of function of RANK display an increased susceptibility to development of pre-neoplastic mammary lesions and mammary tumors (adenocarcinoma, adenosquamous carcinoma and adenomyoepithelioma carcinoma histotypes) following MPA/DMBA treatment [23]. On the contrary, use of the selective pharmacological RANKL inhibitor RANK-Fc reduces mammary epithelial proliferation and attenuates the occurrence of pre-neoplastic lesions and mammary tumors in RANK-transgenic mice and wild-type controls [23]. Transgenic mice overexpressing epidermal growth factor receptor 2 (ErbB2) under the transcriptional control of the mouse mammary tumor virus (MMTV) promoter represent a spontaneous mammary tumor model, which does not require any hormonal exposure for tumorigenesis [81]. Interestingly, RANK-Fc displays anti-tumoral effects even in MMTV-ErbB2 transgenic mice [23].

RANKL and RANK can be both expressed in triple-negative breast cancer (TNBC) [82]. Interestingly, dual expression of RANKL and RANK correlates with a poor prognosis in TNBC patients. In fact, TNBC patients expressing both RANKL and RANK show significantly worse relapse-free survival and overall survival than patients with RANKL-negative RANK-positive TNBCs [82]. These data suggest that RANKL could contribute to spontaneous formation of breast cancer even through hormone-independent mechanisms. Indeed, the presence of RANKL within human mammary tumor epithelium and tumor stroma (e.g. mononuclear cells, fibroblast-like stromal cells) indicates that its activation in breast cancer may be also regulated by mechanisms different from those mediated by progesterone and progestins [23, 76]. Moreover, RANK signaling may promote breast cancer development even through mechanisms other than the well-established induction of cell proliferation. In fact, RANKL/RANK axis favors cell survival protecting DNA-damaged mammary epithelial cells from apoptosis, and controls anchorage-independent growth and self-renewal capacity of tumor-initiating cells [25].

RANKL/RANK system is also involved in epithelial-mesenchymal transition (EMT) [83], which is one of the initial steps in carcinogenesis that promotes the acquisition of stem-like properties and malignant features by epithelial cells (e.g. loss of cell-cell adhesion, enhanced migratory capacity, increased invasive potential, augmented extracellular matrix components, and resistance to apoptosis) [26, 84, 85]. Tsubaki et al. demonstrated that RANKL induces EMT in RANK-expressing normal mammary epithelial cells and breast cancer cells through NF-kB activation and upregulation of Snail and Twist, two transcriptional repressors of the epithelial marker E-cadherin. These molecular events lead to downregulation of E-cadherin and upregulation of mesenchymal markers (e.g. N-cadherin and vimentin), which result in tumor cell migration, invasion and metastasis [26]. Furthermore, there is evidence supporting a potential role of immune system in driving the pro-metastatic behavior of breast cancer cells [86]. Regarding this context, Tan et al. found that RANKL produced by tumor-infiltrating regulatory T cells elicits metastatic spread of mammary cancer cells via RANK signaling [27].

Noteworthy, several studies identified novel RANK isoforms generated through alternative splicing of the *RANK* gene (*TNFRSF11A*: TNF Receptor Superfamily Member 11a), further increasing the functional complexity of RANKL/RANK system in normal and tumor cells [18–20, 87]. Importantly, these isoforms play an important role in the regulation of RANK downstream signalling, mitigating the wild type RANK-mediated promotion of breast cancer initiation, progression and metastasis [18–20]. The RANK isoform RANK-c, which lacks the transmembrane domain and a large portion of the intracellular part of the wild type receptor RANK, has been first detected in breast cancer cells and breast tumors by Papanastasiou et al. [18, 19]. Intriguingly, the authors showed that RANK-c acts as a dominant negative regulator of RANK-dependent NF-kB activation, inhibiting RANK translocation to the cell membrane and the NF-kB-mediated cell survival effect (Fig. 1b). RANK-c expressing breast cancer cells also exhibited lower cell motility and migration rates, indicating a putative role of RANK-c isoform in cytoskeleton remodeling. Moreover, RANK-c expression was found inversely correlated with tumor histological grade and proliferative index, further suggesting a possible role of this isoform as a suppressor of breast cancer progression and metastasis [18, 19]. Sirinian et al. reported that RANK-c is expressed in 3.2% of cases among The Cancer Genome Atlas breast cancer cohort, and its expression is evenly distributed across ER-negative and ER-positive cases. Nonetheless, ER-negative breast cancer cell lines showed an increased RANK/RANK-c ratio compared to ER-positive counterparts. Intriguingly, forced expression of RANK-c in ER-negative breast cancer cell lines was able to counteract NF-kB activation, suppressing aggressive cell properties (e.g. migration, invasion, and colony-forming ability). RANK-c exhibited similar properties in vivo, preventing lung metastases of MDA-MB-231 cells in mice. Moreover, analysis of *RANK-c* transcript levels from primary breast cancer samples showed that RANK-c expression positively correlates with less aggressive disease, as assessed by the absence of distant metastases at the time of diagnosis. At a molecular level, the authors provided evidence that the RANK-c-mediated inhibition of NF-kB activation relies on the interaction with other key molecules, such as TNF receptor-associated factor-2 (TRAF2) and epidermal growth factor receptor (EGFR) [20]. TNF receptor-associated factor (TRAF) proteins are major components of RANK receptor signalling [88, 89]. In presence of RANK-c, TRAF2 preferentially binds to this isoform, excluding RANK from the protein complex. Furthermore, RANK-c has also been shown to act as a negative regulator of EGFR signalling. In fact, RANK-c expressing cells showed impaired EGFR phosphorylation after epidermal growth factor (EGF) ligand stimulation, resulting in inability to activate critical downstream signalling mediators [20] (Fig. 1b). Overall, these data suggest a potential role of RANK-c as a prognostic biomarker in breast cancer, associated with disease severity and metastasis. Nevertheless, clinical studies are needed in order to translate these findings in clinical settings.

A possible correlation between RANK pathway and some members of the human epidermal growth factor receptor (ErbB) family has also been documented [23, 27, 90, 91]. ErbB family consists of four different type I transmembrane growth factor receptor tyrosine kinases (EGFR, HER2, HER3, and HER4), which activate downstream intracellular signaling pathways involved in normal cell development, as well as in human cancer [92, 93]. In fact, EGFR and other members of the ErbB family are often co-expressed in several cancers, contributing to increased cell proliferation and aggressiveness, as well as drug resistance [94–96]. Yi et al. first showed the existence of a strict interaction between RANKL/RANK system and EGFR pathway during osteoclastogenesis, showing that RANKL up-regulates EGFR expression in differentiating osteoclasts. Moreover, inhibition of EGFR blunted the activation of RANKL/RANK signaling pathway and RANKL-dependent osteoclast formation in osteoclast precursor cells, and led to caspase-mediated apoptosis in differentiated osteoclasts [97]. These data highly suggest that EGFR signaling plays a critical role in osteoclast differentiation and survival. Consistent with these findings, RANKL inhibition has been shown to enhance the antineoplastic effects of panitumumab (a fully human anti-EGFR monoclonal antibody) in a murine model of bone metastasis, where it prevented tumor-induced osteolysis and led to a greater reduction in skeletal tumor growth compared to panitumumab alone [98]. Papanastasiou et al. provided evidence of a molecular interaction between RANK and EGFR pathways in primary breast cancer. The authors showed a significant positive correlation between *RANK* mRNA and *EGFR* gene and protein expression in invasive breast cancer samples and breast cancer cell lines, whereas no correlation between RANK and the other ErbB family members was found. Interestingly, breast cancer cells co-expressing RANK and EGFR exhibited a significant enhancement of the EGFR downstream signaling and a higher invasive potential, supporting a synergistic effect of RANK and EGFR at both molecular and cellular level. Moreover, the subgroup of “double positive” breast cancer patients (*RANK*^*hi*^*/EGFR*^*hi*^) displayed a worse clinical outcome, consisting of a reduced overall survival independently of tumor stage and primary lymph node [90]. Different studies also documented the involvement of RANK pathway in ErbB2-positive breast carcinogenesis [23, 27, 91]. ErbB2 (or HER2) is a member of the ErbB receptor tyrosine kinase family; its overexpression is observed in approximately 20% of human breast cancers and correlates with poor prognosis [91]. Indeed, activation of NF-kB - the major downstream mediator of RANK signaling - has been associated with cell survival, proliferation, and invasion, as well as resistance to anti-ErbB2 agents in ErbB2-positive breast cancers [91, 99, 100]. Pharmacological inhibition of RANKL has been shown to decrease spontaneous mammary tumorigenesis, proliferation and metastatic potential in MMTV-ErbB2 transgenic mice [23]. In another study, *MMTV-ErbB2/Rank*^*+/−*^ mice exhibit a remarkable reduction of metastatic rates compared to *MMTV-ErbB2/Rank*^*+/+*^ group [27]. Moreover, the NF-kB-activating protein IKK-α supports ErbB2-induced tumor initiating cells expansion promoting nuclear export of p27, a negative regulator of the G1/S phase transition [101]. Then, NF-kB activity enhances ErbB2-mediated murine mammary tumorigenesis by stimulating tumor angiogenesis [102]. Interestingly, anti-ErbB2 agents can even elicit NF-kB activation, enhancing the oncogene addiction of ErbB2-positive cells to NF-kB [103]. The latter mechanism could provide a rationale for the development of resistance to anti-ErbB2 drugs in ErbB2-positive breast cancer patients [100]. Therefore, the combination of anti-ErbB2 drugs with NF-kB inhibitors [100] or proteasome inhibitors - which prevent NF-kB activation through inhibition of IkB degradation [103] - may represent a novel and more valuable therapeutic approach to treat RANK-expressing ErbB2-positive breast cancers.

Overall, these data strongly encourage further investigation on the potential use of a double pathway inhibition strategy in the subgroup of “double positive” breast cancer patients (RANK-positive and EGFR- and/or ErbB2-positive) through the existing molecules targeting RANKL/RANK pathway and ErbB family members (e.g. denosumab plus anti-EGFR drugs, such as erlotinib or panitumumab; or denosumab plus anti-ErbB2 drugs, such as lapatinib or trastuzumab). Hence, future clinical trials are awaited to assess whether this double inhibition approach may lead to significant advantages.

### Role of RANKL/RANK system in BRCA1 mutation-driven breast tumorigenesis

Approximately 5–10% of breast cancers are hereditary and the vast majority of them are due to germline mutations in *BRCA1* and *BRCA2* tumor suppressor genes [104–106]. *BRCA1* and *BRCA2* encode proteins that cooperate to protect the genome from DNA damage during DNA replication; therefore, loss of these genes causes defective repair of damaged DNA, leading to chromosomal instability and increased cancer susceptibility among mutation carrier patients [107]. Several pre-clinical studies have documented that female sex hormones play an important role in the pathogenesis of *BRCA1*-mediated mammary tumorigenesis. Specifically, BRCA1 is involved in the regulation of both ER and PR, inhibiting the expression of various endogenous estrogen- and progesterone-responsive genes [108–110]. Indeed, progesterone antagonist mifepristone prevents mammary tumorigenesis in *BRCA1*/*p53*-deficient mice [111] and prophylactic salpingo-oophorectomy markedly decreases the risk of developing breast cancer in women with *BRCA1* mutation [112]. Moreover, it has been shown that luteal phase-related levels of estrogen and progesterone are significantly higher in *BRCA1* mutation carriers compared with women not carrying mutation [113]. Given the established role of female sex hormones in the pathogenesis of *BRCA1* mutation-driven breast cancer, different studies investigated whether RANKL/RANK axis could act as a downstream mediator of sex hormones in breast tumorigenesis of *BRCA1* mutation carriers [28, 29, 79]. With this regard, Sigl et al. documented that genetic ablation of *RANK* in basal mammary epithelial cells of mice carrying a *BRCA1;p53* mutation significantly decreases proliferation and markedly abrogates the occurrence of intraepithelial neoplasms and invasive carcinomas [28]. Pharmacological inhibition of RANKL has been found to reduce the development of *BRCA1* mutation-driven pre-neoplastic mammary lesions in mice carrying *BRCA1* mutation. Intriguingly, the human monoclonal antibody denosumab significantly reduces in vitro colony-forming capacity of mammary epithelial progenitor cells from women carrying heterozygous germline *BRCA1* mutations who underwent prophylactic mastectomy. These findings indicate that RANKL/RANK system strictly controls the expansion of *BRCA1*-mutated human mammary progenitor cells. Furthermore, authors identified six single-nucleotide polymorphisms in the locus encoding for human RANK (*TNFRSF11A*), that are significantly associated with breast cancer risk in a wide series of *BRCA1* mutation carriers. Finally, it has also been found that RANKL and RANK are highly expressed in pre-malignant lesions, as well as in breast cancer samples from both *BRCA1* and *BRCA2* human mutation carriers [28]. Consistent with these data, Nolan et al. identified RANK-positive and RANK-negative cells as two distinct subsets of luminal progenitor cells from histologically normal breast tissue of *BRCA1* mutation carriers, demonstrating that RANK-positive progenitors are highly proliferative and more prone to DNA damage. Notably, progesterone-induced proliferation of three-dimensional breast organoids derived from breast biopsies of women carrying *BRCA1* mutation is markedly reduced after exposure to denosumab. Proliferation of mammary epithelial cells - assessed by Ki67 expression - is also significantly reduced in breast biopsies from three *BRCA1* mutation carriers treated with denosumab [29]. Taken together, these data indicate that progesterone-induced RANKL may critically affect *BRCA1*-mutation driven breast tumorigenesis by promoting the expansion of RANK-positive murine and human mammary progenitor cells, which therefore represent a crucial target cell population in *BRCA1* mutation carriers.

### Pitfalls and controversies in detection of RANKL/RANK expression and distribution

In light of the above mentioned findings, RANKL and RANK represent interacting molecules considered as potential therapeutic target in different neoplastic and non-neoplastic diseases. Therefore, their expression and distribution in normal and diseased human tissues are of critical interest in relation to safety and efficacy of drugs targeting the RANKL/RANK pathway. However, immunohistochemical (IHC) methods using a variety of antibodies have shown inconsistencies between the findings comparing the distribution of RANKL and RANK in different tissues, including breast tissue [65, 75, 114, 115]. It is also important to remark that RANKL and RANK expression may vary under different physiological conditions [116], such as the menstrual cycle [75] or the immune response [116, 117]. Nonetheless, it is possible to make some general reflections. In adult tissues, RANKL distribution is more strictly limited to bone (activated osteoblasts), as well as to spleen, peripheral lymph nodes and mammary epithelium [9, 21, 118]. On the other hand, RANK expression occurs in several tissues and is more dependent upon various tissue-specific regulating factors, including progesterone and PTHrP within the mammary epithelium [21, 116–120]. Moreover, reports of the broad RANK protein and mRNA distribution are not consistent with the limited functional role of RANKL/RANK pathway [117], thus highlighting the need for sensitive and specific tools able to detect RANKL and RANK protein expression in both normal and pathologic tissues. This matter is of crucial importance especially for clinical trials evaluating the possible correlation of RANKL and/or RANK tumor expression with clinical outcomes. Indeed, Taylor et al. reported that RANKL detection with IHC methods is relatively straightforward, whereas RANK is a “difficult to detect antigen”. In particular, the ability of IHC methods to detect RANK protein in formalin-fixed paraffin-embedded tissues may be negatively affected by conditions of sample preparation and/or different IHC techniques (e.g. time of fixation, epitope retrieval processes, degree of amplification, different specificity and sensitivity features of the primary antibodies), which are assumed to vary across different laboratories. Indeed, the authors proposed an optimized IHC protocol using well-characterized and highly specific antibodies to properly detect the expression patterns of RANKL and RANK in normal and pathologic tissues and to develop a reproducible assay that could be transferred and compared between laboratories [114]. These observations have a major impact in all studies evaluating the expression of RANKL and/or RANK in human tissues, highlighting that a non-rigorous choice of antibodies or the use of non-validated IHC protocols may lead to misleading findings in RANKL and, particularly, RANK expression.

## Role of OPG in breast tumorigenesis

In skeletal metastases, RANKL/OPG ratio is often increased, with an upregulation of RANKL and a concomitant downregulation of OPG, resulting in osteoclast-mediated bone destruction [44]. Since OPG is a negative regulator of osteoclast maturation and bone resorption [32], early studies focused on the potential use of recombinant OPG to prevent osteolysis related to bone metastasis in breast cancer. Truncated forms of recombinant OPG have been developed, consisting of the N-terminal part of the protein - essential for interaction with RANKL - fused to the Fc domain of human IgG. Interestingly, recombinant OPG has been shown to completely prevent osteolytic metastatic lesions caused by MDA-MB-231 human breast cancer cells in nude and ovariectomized mice [121, 122]. A phase I study demonstrated that the recombinant OPG construct AMGN-0007 leads to a sustained decrease in serum markers of bone resorption when administered to breast cancer patients [123], although development of the compound has been then discontinued due to potential safety risks deriving from an immune response against endogenous OPG [117]. However, other studies showed a more complex role of OPG in breast tumorigenesis [31, 35, 36, 124–127]. In fact, Tan et al. first documented OPG expression in two human breast cancer cell lines, namely MCF-7 and MDA-MB-436 [128]. The expression pattern of OPG has also been assessed by immunohistochemistry in approximately 400 invasive human breast cancer tissue samples: 40% of these tumors showed a strong immunohistochemical OPG expression, which was selectively confined to the tumor cells [35]. A study conducted on 185 patients with primary breast cancer found OPG expression in approximately 46% of cases [78]. Furthermore, OPG expression positively correlates with the presence of ER and PR in human breast tumor samples [76]. Nevertheless, 17beta-estradiol has been shown to suppress OPG production by human ER-positive breast cancer cell lines in a dose-dependent manner [129]. Therefore, the effects of ER activation on OPG expression in breast cancer cells may be different from those observed at the skeletal level under physiological conditions [130]. Given that OPG is not required for normal mammary gland development and lactation [33], its expression may represent a novel mechanism through which tumor cells gain a growth advantage by different molecular mechanisms [31]. In fact, it has been reported that OPG can bind and inhibit TNF related apoptosis-inducing ligand (TRAIL) [131]. TRAIL is a member of the TNF family produced in cancers by invading monocytes, and acts as an inducer of apoptosis in tumor cells upon binding to its death domain-containing cell surface receptors [132] (Fig. 2). Holen et al. showed that OPG can act as an endocrine survival factor in MDA-MB-436 and MDA-MB-231 breast cancer cells by substantially reducing the extent of TRAIL-induced apoptosis [35]. Thus, breast cancer cells could use OPG secretion to gain a survival advantage over the host defenses. However, the relevance of OPG-TRAIL interaction in the context of breast cancer still awaits demonstration in vivo. In fact, it has been shown that MDA-MB-231 human breast cancer cells overexpressing full length OPG display decreased sensitivity to TRAIL-induced apoptosis in vitro, whereas there is a lack of effect in vivo despite the presence of OPG at supraphysiological concentrations [36]. The role of breast cancer cells-derived OPG could be more complex in vivo due to the simultaneous presence of RANKL and TRAIL. Although OPG binds RANKL and TRAIL with the same affinity in vitro [133], the addition of excess RANKL is able to reverse the effect of OPG on TRAIL-mediated apoptosis in human breast cancer cells [125]. Similarly, high levels of RANKL present at a skeletal level - especially in the context of metastatic bone disease [44] - may explain why OPG protects bone microenvironment from breast cancer-induced osteolysis and mitigates intra-osseous tumor growth, whereas it is able to promote primary tumor growth and cancer cells spread to sites out of the bone [134]. However, the strict interactions between TRAIL, OPG, and RANKL in the context of the primary breast tumor still need to be elucidated in vivo. Apart from direct proliferative actions of OPG on breast cancer cells, several studies reported additional mechanisms whereby OPG may exert its tumor-promoting effect in breast cancer. For instance, Cross et al. documented a positive association between endothelial OPG expression and high tumor grade in breast cancers, supporting a potential role of OPG as a pro-angiogenic factor in breast tumor microenvironment [126]. Goswami et al. investigated an in vitro model of angiogenesis, providing evidence for a role of OPG in driving neoangiogenesis in endothelial tube formation [127]. Hence, it is likely that OPG produced either by breast tumor cells or endothelial cells themselves promotes endothelial cell survival and differentiation, inducing angiogenesis and stimulating primary tumor growth [124]. OPG has also been shown to reprogram normal mammary epithelial cells to a tumorigenic state through induction of proliferation and aneuploidy [127]. In addition, Weichhaus et al. demonstrated that OPG stimulates breast cancer cells invasion and metastasis by modulating expression of the proteases Cathepsin D and Matrix Metalloproteinase-2 [135] (Fig. 2). In the same study, the authors also showed that knockdown of OPG in TNBC cells leads to a significant reduction in metastasis in the chick embryo metastasis model [135]. Interestingly, Owen et al. analyzed OPG expression in 127 primary human breast cancer tissues, finding that patients with higher expression of OPG in tumor samples show a significantly poorer overall survival with respect to patients with lower OPG expression [136]. Sarink et al. have recently conducted a large-scale prospective study on 2006 pre- and postmenopausal patients with incident invasive breast cancer participating in the EPIC (European Prospective Investigation into Cancer and Nutrition) cohort. Importantly, the authors showed that higher pre-diagnosis circulating OPG concentrations - assessed by an electrochemiluminescent assay - are associated with a greater risk of breast cancer-specific and overall mortality, especially in ER-positive breast cancer patients [137]. Similarly, Rachner et al. showed that higher OPG serum levels - detected by ELISA - are associated with a significantly higher risk of death from breast cancer in patients with primary, non-metastatic breast cancer. Furthermore, the authors also reported that OPG represents an independent prognostic marker for breast cancer specific survival on multivariate analyses [138]. Nonetheless, these data are in sharp contrast with another study conducted on a large microarray dataset of primary breast cancer patients, which reported that high OPG mRNA levels correlate with longer overall and disease-free survival [139]. Park et al. showed that OPG is not a valuable prognostic factor on multivariate analysis for skeletal-disease free survival, disease-free survival and overall survival in a study based on the analysis of tissue microarrays obtained from 185 patients with primary breast cancer. The authors also found that OPG expression correlates with more favorable tumor clinical and pathologic features, including small tumor size, negative lymph node involvement, and low proliferative index [78]. Overall, these conflicting findings may be related to the diverging effects of OPG expression according to distinct breast cancer subtypes [31] and/or to different methods used for OPG expression analysis in different studies (e.g. quantitative PCR, immunohistochemistry). According to the recent findings from Sarink et al. [137] and Rachner et al. [138], it is also possible that OPG circulating concentrations at diagnosis represent a more informative measure for breast cancer prognosis and mortality than OPG expression in tumor tissue. Further investigations in well-defined patient cohorts (e.g. according to tumor characteristics) are needed to confirm these findings.

**Fig. 2:** Schematic illustration of main OPG sources and actions in breast tumorigenesis. According to most pre-clinical findings, OPG produced by breast cancer and endothelial cells is able to promote tumor growth at the primary tumor site, as well as development of metastatic tumors at extra-skeletal sites, through distinct mechanisms: **a** inhibition of the monocyte-derived apoptosis inducing factor TRAIL, **b** increased expression of some proteases (e.g. cathepsin D, matrix metalloproteinase-2), **c** induction of endothelial cells proliferation and differentiation to form new blood vessels (angiogenesis). Conversely, OPG produced in bone microenvironment can mitigate intra-osseous tumor growth and prevent breast cancer-induced osteolysis by reducing differentiation and activation of mature osteoclasts lining the bone surface. Abbreviations: OPG, osteoprotegerin; TRAIL, TNF related apoptosis-inducing ligand. Adapted from Weichhaus et al., Mol Cancer (ref. [31])

Finally, OPG produced by breast cancer cells appears to contribute to tumor growth and progression at the primary tumor site, while acting as a protective factor in bone microenvironment by preventing breast cancer-induced bone loss and reducing intra-osseous tumor growth. Nevertheless, most of these data derive from observations in vitro and further studies are warranted to confirm whether OPG exerts the same effects in vivo.

## Influence of RANKL/RANK/OPG system on bone metastasis in breast cancer

Breast cancer represents a neoplasm with high propensity to spread to bone; in fact, about 70% of patients with advanced breast cancer develop bone metastases [140]. Of note, skeletal invasion of breast cancer cells is usually associated with osteolytic lesions [141], which lead to sustained bone resorption and skeletal-related events (SREs), defined as pathological fractures, hypercalcemia, spinal cord compression, or bone pain [142]. RANKL/RANK/OPG system may have an important role in promoting migration of breast cancer cells to the bone and their subsequent metastatic behavior [23, 24, 26, 135, 143]. In fact, RANKL has been reported to accelerate the migration and metastasis of RANK-expressing cancer cells [24]. High levels of RANK in tumor specimens from patients with primary breast cancer have been correlated with poor prognosis, higher risk to develop bone metastases, and shorter skeletal disease-free survival [139]. Moreover, an high concordance in RANK expression between bone metastasis and corresponding breast primary tumor has been also reported [77]. A recent retrospective analysis on a cohort of 509 patients with primary, non-metastatic breast cancer (median follow-up: 8.50 years; median age of participants: 60 years) found that RANKL serum levels were significantly higher in patients with disseminated tumor cells in the bone marrow, as well as in patients who developed bone metastases. Moreover, patients within the highest quartile of RANKL showed a significantly increased risk of developing bone metastases compared to those in the lowest quartile [138].

The exact role of OPG within the bone metastatic niche in breast cancer still remains controversial [31, 122, 124, 135, 144–146]. Neville-Webbe et al. showed that bone marrow stromal cells isolated from breast cancer patients are able to produce OPG at levels that are sufficient to protect breast cancer cells from TRAIL-induced apoptosis, supporting a role of bone-derived OPG in promoting survival of breast cancer cells within the bone metastatic niche [144]. However, Ottewell et al. found that recombinant OPG markedly counteracts growth of dormant MDA-MB-231 cells at the skeletal level in a murine model of disseminated breast cancer cells, thus preventing development of bone metastases [122]. Chanda et al. investigated the effects of sustained OPG-Fc expression using a recombinant adeno-associated viral vector in a mouse model of osteolytic breast cancer, finding a significant reduction in skeletal tumor growth and bone loss, despite no effects on long-term survival [145]. Moreover, a conditionally replicating adenovirus (CRAd) characterized by a shortened OPG-Fc reduced tumor burden in the bone and osteoclast formation more effectively than an unarmed CRAd in a murine model of osteolytic bone metastases of breast cancer [146].

As cancer cells home to bone, favorable interactions between these cells and bone microenvironment are essential for the initiation of osteolytic metastasis, according to the “seed and soil” hypothesis [147]. In this context, impaired regulation of RANKL/RANK/OPG system and excessive osteoclast-induced bone resorption have been shown to play an important role in promoting bone metastasis in certain malignant diseases, including breast cancer [148]. Breast tumor cells can secrete PTHrP and other soluble mediators (e.g. TNF-α, IL-1, IL-6, IL-8, M-CSF) able to promote osteoclastogenesis and osteolytic lesions through RANKL upregulation by osteoblasts and stromal cells [149, 150]. PTHrP can also decrease OPG levels from osteoblasts [151], further upregulating RANKL-to-OPG ratio in skeletal metastases [44]. Therefore, osteoclastic resorption gives rise to increased release of TGF-β (transforming growth factor-β) and other soluble factors from the bone matrix, which promote increased proliferation of cancer cells and enhance PTHrP production [150, 152]. In turn, PTHrP stimulates osteoblasts and stromal cells to secrete RANKL, which drives osteoclast activation and further release of TGF-β from the bone [150, 151]. The complex cross-talk between breast cancer cells and bone microenvironment is thereby responsible for a detrimental “vicious cycle”, which ultimately favors metastatic tumor promotion, progression and bone destruction, with the establishment of de novo bone metastasis and severe clinical morbidities [44].

## Therapeutic perspectives in humans: targeting RANKL/RANK/OPG system for prevention and treatment of breast cancer

As previously discussed, RANKL accelerates the migration and metastasis of RANK-expressing cancer cells [24] and acts as the final effector of osteoclastogenesis in the vicious cycle of bone destruction in metastatic bone disease [150]. Thus, inhibition of RANKL may potentially counteract migration of RANK-positive cancer cells and make the bone less attractive for these cells, preventing and reducing tumor outgrowth in the skeleton. This phenomenon could rely, at least in part, on the fact that inhibition of RANKL is able to curb the direct effect of RANKL on RANK-expressing cancer cells [23, 86]. In humans, inhibition of RANKL/RANK system can be obtained from the use of the human monoclonal antibody denosumab, that specifically inhibits RANKL and blocks its binding to RANK. Denosumab is currently used in clinical settings for the treatment of women at high risk for bone fractures, such as postmenopausal women with osteoporosis and patients with non-metastastic breast cancer on aromatase inhibitors therapy [153, 154]. High dose denosumab (120 mg every 4 weeks) has recently become a standard of care, in addition to chemotherapy, in patients with bone metastatic breast cancer [155], where it has been shown superior to bisphosphonates in delaying or preventing SREs [142, 156–158]. The difference between denosumab and bisphosphonates in SREs prevention may depend on the distinct mechanisms of action of the two agents. In fact, bisphosphonates act only on mature and active osteoclasts, whereas inhibition of RANKL prevents survival, activation and differentiation of osteoclasts from their precursor cells, leading to a total lack of osteoclasts in treated bone [159]. However, no significant differences in overall survival have been observed among patients with bone metastatic breast cancer receiving either denosumab or zoledronate [156].

In agreement with pre-clinical findings [23, 46], accumulating evidence highlights RANKL/RANK pathway as a potential therapeutic target not only in bone metastasis management, but even in breast cancer prevention and adjuvant clinical settings [86]. In fact, ongoing clinical trials are evaluating if denosumab is able to prevent the development of bone metastasis and disease recurrence in the adjuvant phase of breast cancer treatment [86]. Early promising data have been shown from the ABCSG-18 study, an ongoing randomized phase III trial recruiting postmenopausal women with early-phase hormone receptor-positive breast cancer treated with aromatase inhibitors as adjuvant therapy and randomly assigned to receive either placebo or denosumab 60 mg every 6 months (ClinicalTrials.gov identifier: NCT00556374). Patients receiving denosumab have shown a significant delayed time to first clinical fracture (primary endpoint of the study) compared with placebo group. Importantly, reduction in fracture risk was irrespective of age and baseline bone mineral density [160]. According to current evidence, zoledronate or six monthly denosumab for the entire duration of aromatase inhibitors therapy represents the standard of care in postmenopausal women receiving aromatase inhibitors, aimed at preventing bone loss associated with the adjuvant hormonal therapy. Of note, denosumab is recommended when fracture prevention is the priority, whereas zoledronate when breast cancer recurrence is the major concern [154]. To date, adjuvant bisphosphonate treatment in breast cancer has been found to reduce disease recurrence and improve disease-free survival and overall survival only in postmenopausal settings [157, 161]. However, there is still a lack of knowledge about the different impact of bisphosphonates and denosumab on disease recurrence and overall survival among patients with early and advanced non-metastatic breast cancer. Preliminary results from ABCSG-18 suggest a significant improvement in disease-free survival among patients receiving denosumab with respect to placebo group after 5 and 8 years of follow-up [160, 162]. As a consequence, denosumab may be offered to all postmenopausal women with hormone receptor-positive breast cancer on aromatase inhibitors, not only for aromatase inhibitor-associated bone loss and bone fractures prevention, but even for adjuvant purposes, including improvement in disease-free survival [163]. However, these promising results are in contrast with those observed in the D-CARE trial (ClinicalTrials.gov identifier: NCT01077154), a randomized phase III placebo-controlled study which has been recently terminated. D-CARE trial had the primary objective to evaluate whether 5-year denosumab administration (at higher doses compared with those used in the ABCSG-18 study, namely: 120 mg every 4 weeks for 6 months, then 120 mg every 3 months) is superior to placebo in improving disease-specific outcomes (bone-metastasis free survival, disease-free survival and overall survival) in women with early-stage breast cancer receiving optimal loco-regional and standard of care systemic (neo)adjuvant therapy. After a median follow-up of 67 months, denosumab showed improvement in time to bone metastasis as first recurrence, but it did not improve bone-metastasis free survival, disease-free survival and overall survival in all the study groups (including the subset of postmenopausal patients) [164]. These opposing results may be partly explained by the different features of the subjects recruited in D-CARE and ABCSG-18 trials. In fact, D-CARE study enrolled a more heterogeneous population, consisting of both pre- and postmenopausal breast cancer patients. Noteworthy, patients in D-CARE trial were also at high risk of disease recurrence, as defined by lymph node-positive disease (assessed by biopsy evaluation) and/or tumor size > 5 cm (T3) or locally advanced disease (T4). On the other hand, ABCSG-18 trial has recruited only postmenopausal women with histologically confirmed non-metastatic hormone receptor-positive breast cancer receiving treatment with adjuvant aromatase inhibitors [160, 162]. Therefore, long-term data from ABCSG-18 study will be helpful to further assess the effects of denosumab on additional outcomes, such as bone-metastasis free survival and overall survival.

Moreover, clinical trials are deemed necessary to evaluate disease recurrence and overall survival in pre- and postmenopausal women with early hormone sensitive breast cancer on adjuvant hormonal therapy (tamoxifen, aromatase inhibitors) receiving either denosumab or zoledronate to prevent cancer treatment-induced bone loss. Additional data on the role of denosumab as a potential anti-tumor agent in breast cancer are expected from PERIDENO (ClinicalTrials.gov identifier: NCT03532087), a prospective randomized phase II study investigating the impact of (neo)adjuvant denosumab on systemic immunity and local immune microenvironment in postmenopausal patients with early breast cancer. It is also important to note that RANK expression has been found in a subset of TNBCs [82]. With this regard, an upcoming randomized phase II neoadjuvant clinical trial (GeparX, ClinicalTrials.gov identifier: NCT02682693) is recruiting patients with hormone receptor-negative primary breast cancer in order to assess whether administration of denosumab (120 mg every 4 weeks for 6 cycles) as an add-on neoadjuvant treatment is able to increase pathological complete response rate and improve outcome in relation to RANK tumor expression.

As previously mentioned, pre-clinical studies have shown that denosumab reduces mammary epithelial and progenitor cells proliferation in patients with *BRCA1* mutation [28, 29, 165]. Therefore, pharmacological inhibition of RANKL may be also considered as a novel, promising targeted approach in *BRCA1* mutation carriers, aimed at preventing breast cancer initiation. In particular, large randomized clinical trials on *BRCA1* mutation carriers are needed to ascertain if denosumab is able to reduce breast cancer risk when associated with active surveillance in primary prevention. In this context, denosumab could be considered as a useful therapeutic strategy in premenopausal settings, aimed at delaying the need for bilateral prophylactic mastectomy and counteracting the bone loss after bilateral prophylactic salpingo-oophorectomy. With this regard, the pilot study BRCA-D (Trial ID: ACTRN12614000694617) is recruiting pre-menopausal women carrying a *BRCA1* or *BRCA2* mutation to establish if denosumab (120 mg monthly for 3 months) affects proliferation - assessed by Ki67 expression - in the breast epithelium of such individuals. Since RANK expression has been detected in a relevant proportion of cancers arising in *BRCA1* mutation carriers [79], it will be also critical to investigate if RANKL inhibition can abrogate breast cancer progression at the early stages of tumorigenesis and/or if it offers significant advantages as add-on treatment option to adjuvant hormonal therapy in reducing the risk for contralateral breast cancer [166]. It is worth to note that RANKL expression is markedly upregulated in postmenopausal women, resulting in augmented bone resorption and increased risk for osteoporosis [167]. In turn, RANKL upregulation in bone microenvironment may play direct effects on RANK-expressing breast cancer cells. In light of these data, RANKL inhibition may be potentially beneficial especially for postmenopausal women, including those carrying *BRCA1* mutation.

In conclusion, the therapeutic potential of targeting OPG is still under debate. Indeed, the therapeutic use of recombinant OPG for prevention of bone metastasis in breast cancer is currently strongly limited by the lack of knowledge on the exact role of OPG in human breast tumorigenesis. Importantly, OPG can no longer be considered as a factor acting solely within the bone microenvironment in breast cancer. Hence, caution should be used in the development of systemic therapies aimed at increasing OPG levels in patients with breast cancer. Moreover, the beneficial effects showed by denosumab in delaying or preventing SREs in bone metastatic breast cancer [142, 156–158] is likely to have overwhelmed the clinical research on the use of recombinant OPG for prevention of osteolysis associated with metastatic bone disease, as well as for prevention of bone metastatic disease itself. In fact, the therapeutic use of OPG in breast cancer has no longer been studied, since the phase I study evaluating the skeletal effects of the AMGN-0007 compound has been interrupted [117]. In light of our current knowledge, we believe that the use of recombinant OPG in the future may be limited to patients with bone metastatic breast cancer, which could benefit from its administration in terms of morbidity and mortality. However, future studies are needed to evaluate the real feasibility and efficacy of therapeutic strategies for localized delivery of OPG to the bone (e.g. gene therapy), aimed at inhibiting osteolysis and bone loss in patients with bone metastatic breast cancer.

## Concluding remarks and future directions

A growing body of evidence points toward a critical involvement of RANKL/RANK pathway in breast cancer initiation and progression through different mechanisms, such as increased proliferation and survival of mammary epithelial cells, enhanced MaSCs expansion, and induction of EMT. At a molecular level, expression of RANKL and RANK within mammary gland is mainly regulated by progesterone. Thus, RANKL/RANK system may represent one of the key factors linking progesterone and progestins to increased breast cancer risk in women. However, the existence of hormone-independent mechanisms controlling mammary RANKL and RANK expression has also been postulated. RANKL and RANK expression has been documented in different human breast cancers subtypes, including hormone receptor-positive cancers, TNBCs and *BRCA*-deficient cancers. Moreover, RANKL- and/or RANK-positive breast cancers have been associated with a poor prognosis in different clinical studies. To date, targeting RANKL represents a valid therapeutic approach to prevent and manage SREs in the context of bone metastatic breast cancer. Furthermore, a series of pre-clinical studies demonstrated that RANKL inhibition reduces proliferation of mammary epithelial cells and MaSCs, besides attenuating the occurrence of pre-neoplastic lesions and mammary tumors. Based on pre-clinical findings, RANKL inhibition may play also a central role in prevention of disease recurrence and bone metastases in the context of established breast cancer. Nonetheless, whether denosumab may have a place in breast cancer prevention and treatment among the subpopulation of RANK-expressing early breast cancer patients is still an open question. It will be also important to evaluate if a large spectrum of breast cancer patients may benefit from denosumab, or if its use is substantially limited to specific age and/or breast cancer subtypes.

Overall, results from ongoing studies and future large randomized clinical trials are awaited to assess the potential use of denosumab as an anti-tumor agent in different breast cancer settings, namely: a) as a disease-modifying agent in hormone receptor-positive breast cancer patients on adjuvant hormonal therapy, which would be beneficial even for prevention of cancer treatment-induced bone loss, b) as a disease-modifying agent in patients with TNBC and ErbB2-positive breast cancer, c) as an add-on adjuvant therapy in *BRCA1* mutation carriers for the treatment of established breast cancer and/or prevention of contralateral breast cancer, d) as a novel chemoprevention approach in *BRCA1* mutation carriers, aimed at reducing breast cancer risk, delaying the need for bilateral prophylactic mastectomy and counteracting the prophylactic oophorectomy-induced bone loss. As extensively discussed, RANKL/RANK system is a key paracrine effector of progesterone signaling on breast epithelium and repeated proliferative cell response elicited by progesterone-RANKL axis can represent a risk factor for breast cancer. In this context, young premenopausal women with high risk for breast cancer may become a potential target group to study the effectiveness of denosumab in preventing breast cancer.

Finally, data on the exact role of OPG in tumorigenesis and metastatic process, as well as its prognostic value in human breast cancer are still under debate. According to pre-clinical findings, effects of OPG in breast cancer appear to vary depending on its site of action. Indeed, interaction of OPG with breast cancer cells can lead to tumor growth and progression through different mechanisms. However, in vitro and in vivo studies on the role of OPG in breast tumorigenesis are controversial: in fact, in vitro studies suggest a role of OPG in promoting primary tumor growth and progression, whereas there is a lack of effect in vivo. These conflicting findings may depend on the complex interactions between OPG, TRAIL and RANKL in vivo. On the other hand, most pre-clinical studies suggest a protective role of OPG against tumor growth and osteolysis within the bone metastatic niche in breast cancer. Nonetheless, caution should be taken in translating pre-clinical findings on the role of OPG in breast tumorigenesis to humans, as well as in development of systemic therapeutic strategies aimed at increasing OPG levels in patients with bone metastatic breast cancer. Therefore, future studies are required to better elucidate the role of OPG in breast cancer initiation and progression in vivo, and to subsequently investigate the potential efficacy of therapeutic strategies targeting OPG in different breast cancer settings.
